# Effect of Stellate Ganglion Block Combined with Lidocaine at Different Concentrations for Preemptive Analgesia on Postoperative Pain Relief and Adverse Reactions of Patients Undergoing Laparoscopic Cholecystectomy

This article has been retracted.

**DOI:** 10.1155/2022/6027093

**Published:** 2022-04-11

**Authors:** Zhen Wang, Jiao Yu, Tongxiang Niu, Zhijiang Dong, Zhijun Yin

**Affiliations:** ^1^Department of Hepatobiliary Surgery, Tianjin Jinnan Hospital, 1 Anrong Road, Jinnan District, Tianjin, 300052, China; ^2^Department of Hepatobiliary Surgery, Tianjin Medical University General Hospital, Tianjin 300120, China; ^3^Department of Anesthesiology, Tianjin Jinnan Hospital, Tianjin 300052, China

## Abstract

**Objective:**

To explore the effect of stellate ganglion block (SGB) combined with lidocaine at different concentrations for preemptive analgesia on postoperative pain relief and adverse reactions of patients undergoing laparoscopic cholecystectomy (LC).

**Methods:**

Ninety patients undergoing LC in our hospital from June 2019 to June 2020 were selected as the subjects and were randomly divided into group A (30 cases), group B (30 cases), and group C (30 cases), all patients received SGB, and 10 mL of lidocaine at concentrations of 0.25%, 0.5%, and 0.75% was, respectively, administered to patients in groups A, B, and C, so as to compare the analgesic effect, adverse reactions, and clinical indicators among the three groups.

**Results:**

At *T*_1_ and *T*_2_, group C obtained obviously lower NRS scores than groups A and B (*P* < 0.001); compared with groups A and B, group A had obviously higher onset time (*P* < 0.001) and significantly lower duration (*P* < 0.001); no obvious differences in the hemodynamic indexes among the groups were observed (*P* > 0.05); group C obtained obviously higher BCS score than groups A and B; and the total incidence rate of adverse reactions was obviously higher in group C than in groups A and B (*P* < 0.05).

**Conclusion:**

Performing SGB combined with 0.5% lidocaine to patients undergoing LC achieves the optimal analgesic effect; such anesthesia plan can effectively stabilize patients' hemodynamics, present higher safety, and promote the regulation of the body internal environment. Further research will be conducive to establishing a better anesthesia plan for such patients.

## 1. Introduction

Hepatobiliary diseases are relatively common in China, especially represented by gallstones due to cholecystitis, which have become one of the major diseases that jeopardize people's health [1]. Cholecystitis triggers symptoms of nausea and epigastric pain, while gallstones trigger symptoms such as biliary colic and vomiting. Relevant published works have pointed out a higher incidence in women than in men and a higher incidence at older ages [2]. Naoko et al. [3] et al. stated that the incidence of gallstones in the population was about 6.59%, and the incidence over the age of 40 was about 10.15%. In addition, with the aging of the domestic population, changes in the diet structure and improved diagnosis and treatment techniques, the incidence and detection rates of gallbladder diseases also show an increasing trend, which can seriously affect people's quality of life (QOL) [4]. Abdelrahman [5] et al. reported that it has been more than 100 years since German surgeons completed the first cholecystectomy in 1882, which greatly contributed to the development of biliary surgery. With the continuous improvement of medical technology and the progress of science and technology, laparoscopy emerges as the times require. Matteo [6] et al. mentioned that laparoscopy was developed in 1991 in China and is now popularized all over the country. And now, laparoscopic cholecystectomy (LC) has become the “gold standard” for the treatment of benign diseases of the gallbladder because of its unique advantages such as low cost, little surgical trauma, and fast recovery, and it is accepted by a wide range of patients and physicians [7].

Despite its significant therapeutic effects, LC requires the establishment of a CO_2_ pneumoperitoneum, is highly irritating, and may easily cause hemodynamic changes in patients during the perioperative period due to the influence by surgical position and general anesthesia [8]. At the same time, most patients still suffer from postoperative pain due to factors such as punctured holes in the abdominal wall and visceral traction, thus affecting their postoperative recovery. Stellate ganglion block (SGB) belongs to the cervical sympathetic block, which can achieve the effect of analgesia by blocking the central nerve action as well as the peripheral nerve fiber action, gradually becoming the main analgesia therapy in recent years [9]. And applying lidocaine in this treatment modality results in a more desirable analgesic effect. In addition, SGB can not only regulate hypothalamic and peripheral nerve block and reduce the stress response and pain of patients but also affect the immune system of patients while protecting the brain, so it is frequently applied in the clinic. Study by De la Gala [10] and others have confirmed that SGB combined with lidocaine at a dose of 10 mL and a 0.5% concentration has achieved significant results in abdominal surgery. But further research is required to explore whether increasing or decreasing lidocaine concentration can improve the preemptive analgesic effect and prolong the analgesia time. Based on this, this study provides more evidence for subsequent clinical treatment by exploring the analgesic efficacy and safety of SGB combined with lidocaine at different concentrations for patients undergoing LC, with the results reported as follows:

## 2. Materials and Methods

### 2.1. General Data

Ninety patients undergoing LC in our hospital from June 2019 to June 2020 were selected as the subjects and were randomly divided into group A (30 cases), group B (30 cases), and group C (30 cases); all patients received SGB, and 10 mL of lidocaine at concentrations of 0.25%, 0.5%, and 0.75% was, respectively, administered to patients in groups A, B, and C. The study met the World Medical Association Declaration of Helsinki [11].

### 2.2. Enrollment of Study Subjects

The following are the inclusion criteria: (1) the patients underwent selective surgery; (2) the patients had stable blood pressure and heart rate under monitoring before surgery; (3) the American Society of Anaesthesiologists (ASA) [12] class was I-II; (4) the patients had gallstone (benign) and gallbladder polyp with chronic cholecystitis according to the finding of ultrasound examination and received LC in our hospital; and ⑤ the patients did not suffer from diabetes and hyperlipidemia before surgery.

The following are the exclusion criteria for the patients: (1) complicated with severe lesion in the heart, liver, kidney, lung, and other organs; (2) presence of hearing or seeing disorders; (3) taking sedative medications or antidepressant medications, etc., before or during the trial; (4) presence of severe psychological illness; (5) complicated with central nervous system disease; (6) known allergy or suspected allergy to amide drugs; (7) complicated with infectious diseases; and (8) history of alcohol and medication dependence.

### 2.3. Methods

#### 2.3.1. Anesthesia Methods

The vein passage was established before anesthesia, the heart rate, blood pressure, and pulse oxygen saturation were monitored with the patient monitor (manufacturer: IVY Biomedical systems, Inc.; model: 3150), and oxygen inhalation was performed to patients with the oxygen mask at the same time. Thirty minutes before surgery, 10 mL of lidocaine (manufacturer: Xi'an Disai Biological Pharmaceutical Co., Ltd.; NMPA approval no. H61020713; specification: 20 mL: 400 mg) was administered to patients at the root of the right anterior tubercle of the transverse process of the sixth cervical spine (C6), the concentrations of lidocaine for groups A, B, and C were, respectively, 0.25%, 0.5%, and 0.75%, and if patients presented symptoms of the Horner syndrome [13] such as facial hypohidrosis on the block side, palpebral fissure becoming smaller, ptosis of upper eyelid, enophthalmos, and miosis, it was regarded as the signs of markedly effective SGB.

#### 2.3.2. Anesthesia Induction

Anesthesia induction was performed to all patients with the sequence of administration being 0.002~0.004 mg/kg of fentanyl (manufacturer: Langfang Branch, China National Pharmaceutical Industry Corporation Ltd.; NMPA approval no. H20123298; specification: 10 mL : 0.5 mg), 0.3 mg of etomidate (manufacturer: Jiangsu Hengrui Medicine Co., Ltd.; NMPA approval no. H32022379; specification: 10 mL : 20 mg), and 0.6 mg of rocuronium (manufacturer: North China Pharmaceutical Co., Ltd.; NMPA approval no. H20103495; specification: 2.5 ml : 25 mg); tracheal intubation was performed within 60 s; after that, the anesthesia machine (manufacturer: Draeger Medical Equipment (Shanghai) Co., Ltd.; specification: Fabius2000) was connected to give anesthesia support with the tidal volume set as 7 mL/kg.

#### 2.3.3. Anesthesia Maintenance

For anesthesia maintenance, 2~3 *μ*g of propofol (manufacturer: Guangdong Jiabo Pharmaceutical Co., Ltd.; NMPA approval no. H20010368; specification: 10 mL : 100 mg∗5 bottles/box∗40 boxes) was given via plasma target-controlled infusion until 5 min before surgery, and 0.1~0.15 *μ*g/(kg·min) of remifentanil (manufacturer: Yichang Humanwell Pharmaceutical Co., Ltd.; NMPA approval no. H20030200; specification 5 mg) was administered till the end of surgery. To avoid too light anesthesia or incomplete analgesia, the bispectral index was maintained between 40 and 60, the patients' respiratory rate was adjusted, the end tidal carbon dioxide partial pressure was maintained between 30~40 mmHg to avoid CO_2_ detention, and muscle relaxant could be added during surgery according to the surgery time and anesthesia depth.

### 2.4. Observation Indicators

Postoperative 12 h, 24 h, and 48 h were, respectively, set as *T*_0_, *T*_1_, and *T*_2_, and the pain degree of patients in the three groups at different time points was evaluated by referring to the Numerical Rating Scale (NRS) [14]. The maximum score of the scale was 10 points, with higher scores indicating more intense pain.

The onset time (start of administration to the appearance of markedly effective features of SGB) and duration (the duration of markedly effective features of SGB) were compared among the three groups.

The electrocardiograph (manufacturer: Beijing Choice Electronic Tech Co., Ltd.; model: MD100) and pulse oximeter (manufacturer: Shenzhen Creative Industry Co., Ltd.; model: PC-68A) were used to record the hemodynamic indexes of patients in the three groups before SGB and 5 min after SGB, including heart rate (HR), systolic blood pressure (SBP), diastolic blood pressure (DBP), and oxygen saturation (SaO_2_).

The comfort of patients in the three groups was evaluated by Bruggrmann Comfort Scale (BCS) [15], with 0 point indicating continuous pain; 1 point indicating painless without movement, severe pain while breathing deeply or coughing; 2 points indicating painless without movement, mild pain while breathing deeply or coughing; 3 points indicating painless when breathing deeply; and 4 points indicating painless when coughing. On a scale of 0-4 points, higher scores indicated higher degree of comfort.

Unified follow-up was carried out to patients by means of telephone, WeChat, interview, etc.; the frequency was 4 times per week for a total of 2 weeks, so as to record the incidence rates of adverse reactions (pharyngeal discomfort, hoarseness, abnormal sensation in the upper limbs, and dizziness) in patients of the three groups in detail.

### 2.5. Statistical Processing

The experimental data were statistically analyzed and processed by SPSS21.0, the picture drawing software was GraphPad Prism 7 (GraphPad Software, San Diego, USA), the enumeration data were examined by *X*^2^ test and expressed by *n*(%), the measurement data were examined by a *t*-test and expressed by $\bar{\text{x}}\pm s$, and differences were considered statistically significant at *P* < 0.05.

## 3. Results

### 3.1. Clinical Data

No significant differences in gender, mean age, mean height, BMI, surgery time, ASA class, educational degree, complicating disease, household economy, and place of residence of patients in the three groups were observed (*P* > 0.05), presenting comparability. See Table 1.

### 3.2. NRS Scores

At *T*_1_ and *T*_2_, the NRS scores were obviously lower in group C than in groups A and B (*P* < 0.001). See Figure 1.

### 3.3. Onset Time and Duration

Compared with groups B and C, group A presented obviously higher onset time and lower duration (all *P* < 0.001). See Table 2.

### 3.4. Hemodynamic Indexes

No obvious differences in the hemodynamic indexes among the groups were observed (*P* > 0.05). See Table 3.

### 3.5. BCS Scores

Compared with groups A and B, group C obtained obviously higher BCS score (*P* < 0.001). See Figure 2.

### 3.6. Adverse Reaction Rates

Compared with groups A and B, group C presented obviously higher total incidence rate of adverse reactions (*P* < 0.05). See Table 4.

## 4. Discussion

As an analgesic specific modality, SGB is widely used in preemptive analgesia, which can further relieve the hyperfunction and excessive tension of stellate ganglion by reversibly blocking the ganglion, making the preganglionic and postganglionic fibers temporarily lose function, thus easing pain, improving blood circulation, regulating endocrine and cardiovascular systems, and achieving the purpose of treating diseases [16]. In addition, the stellate ganglion is a cervical sympathetic ganglion, which is merged by the inferior cervical ganglion from C_3-7_ with the first thoracic sympathetic ganglion and sometimes including *T*_2_ and middle cervical ganglia. Relevant published works have pointed out that SGB can improve patient tolerance to surgical trauma and ensure perioperative safety and treatment efficacy [17]. The indications for SGB are broad, including systemic disorders (myasthenia gravis), head disorders (cerebral vascular spasm), and eye disorders (cataracts). Bataineh [18] et al. demonstrated that continuous SGB was effective in reducing the occurrence of cerebral vascular spasm in patients undergoing intracranial aneurysm intervention. The study by Offiah [19] et al. confirmed that left SGB could reduce perioperative sympathetic activity in patients undergoing coronary artery bypass grafting, which had a promoting effect on balance of autonomic function. Due to perforating injuries to the abdominal wall, traction from the viscera and peritoneum, and persistent stimulation of the nerve endings of the peritoneum by H^+^ derived from CO_2_ uptake by the peritoneum, laparoscopic resection causes severe pain sensation to patients [20]. The main characteristic of laparoscopic gallbladder surgery is that CO_2_ pneumoperitoneum is constructed intraoperatively, so that the patients' intra-abdominal pressure and airway pressure rise, and with CO_2_ being absorbed into blood, the abdominal cavity microenvironment will be changed, which will then lead to the release of plasma catecholamines and other active substances and triggers stress responses. In addition, surgery, as a noxious stimulus, triggers peripheral tissues to generate and release of a variety of chemokines and cytokines that, while engaging in the activation and modulation of receptors, produce painful feelings for patients. Studies have shown that lidocaine administered to patients is not only effective in reducing pain sensation but also beneficial to patient outcomes, and many reports have confirmed that SGB combined with lidocaine achieves significant preemptive analgesia effect [21]. In this study, lidocaine at the same dose but at different concentrations was applied in groups A, B, and C, in which NRS scores at *T*_1_ and *T*_2_ in group C were significantly lower than those in groups A and B (*P* < 0.001), indicating that, at the same dose, SGB combined with lidocaine was effective in reducing pain sensation in patients and that higher lidocaine concentrations resulted in better analgesia. Gao [22] et al. stated that the minimum anesthetic concentration of a local anesthetic is related to the thickness of nerve fibers, and sometimes only very low concentrations can act as a block. And the study results showed that compared with groups B and C, group A presented obviously higher onset time and lower duration (all *P* < 0.001), proving that 0.25% lidocaine had a significantly faster onset time and some block effect, although its duration was not as long as that in the other two groups.

Patients experience a series of operations, such as artificial pneumoperitoneum, tracheal intubation, and cholecystectomy in the perioperative period, which, combined with a great psychological burden, can very easily cause the body to have an intense stress response, thus altering endocrine function, resulting in dramatic hemodynamic fluctuations, leading to the occurrence of reactions such as increased heart rate and higher blood pressure. Katsumori [23] et al. pointed out that hemodynamic stability to some extent reflects the intensity of stress response, which indirectly suggests perioperative safety. And the study results showed no obvious differences in the hemodynamic indexes among the groups (*P* > 0.05), suggesting that lidocaine at different concentrations caused little impact on patients' hemodynamics and had higher safety. SGB also has less effect on the body hemodynamic indicators and enables more stable circulatory function changes; the reason is that SGB can inhibit the hypothalamic-pituitary-adrenal axis, reduce the release of catechol and other substances, alleviate the stress response, and thus maintain the body hemodynamic stability. Meanwhile, compared with those in groups A and B, the BCS score was obviously higher in group C (*P* < 0.05), demonstrating that at the same dose, the higher the concentration of anesthesia, the lower the pain sensation, and the higher the level of comfort. However, it was found that after the administration of lidocaine, some patients were prone to multiple adverse effects, such as dizziness, pharyngeal discomfort, and hoarseness, and the risk of adverse effects was mostly related to the concentration of lidocaine applied, the higher the concentration, the higher the risk of adverse effects. Hu [24] et al. confirmed that the related adverse effects caused by local anesthetics were positively correlated with the dose, in addition to the operational technique. The results of the study indicated that group C presented obviously higher total incidence rate of adverse effects than groups A and B (*P* < 0.05), implying that higher concentration resulted in lower safety, which is comparable to the results of Naris and Chulabhorn [25], who reported that 0.4% and 1% lidocaine combined with SGB were effective in the treatment of migraine, but there was a trend towards increased complications with high concentrations of lidocaine. There are deficiencies of the study: not sufficient sample size was included in this clinical study due to the limited observation time, which caused bias in the results; scales were still the method for clinical evaluation, so there must be certain subjectivity and intentions when patients were answering the questions, which might affect the final results of the clinical trial to some extent; in addition, SGB was also applied in this study, but whether SGB technique will cause postoperative cognitive impairment in patients and the mechanism of higher incidence of adverse effects at higher concentration need further study. Therefore, future research should expand the sample size, refine the clinical experimental design, and optimize the evaluation indexes, so as to obtain more precise conclusions.

In conclusion, SGB combined with lidocaine achieves significant preemptive analgesia effect, lidocaine at three concentrations produces no obvious impact on vital signs, but different concentrations of lidocaine presents different analgesic effects, resulting in better analgesia in group B than in group A and better safety in group B than group C. Therefore, 0.75% lidocaine is more suitable for later clinical relevant treatment.

## Figures and Tables

**Figure 1:** NRS scores ($\bar{x}\pm s$). The figure shows the comparison of NRS scores at different time points among the three groups, the horizontal axis indicated *T*_0_, *T*_1_, and *T*_2_, and the vertical axis indicated the NRS score (points). At *T*_0_, *T*_1_, and *T*_2_, the NRS scores of group A were, respectively, 8.53 ± 0.51, 7.47 ± 0.51, and 5.50 ± 0.51. At *T*_0_, *T*_1_, and *T*_2_, the NRS scores of group B were, respectively, 8.50 ± 0.51, 6.57 ± 0.50, and 3.47 ± 0.51. At *T*_0_, *T*_1_, and *T*_2_, the NRS scores of group C were, respectively, 8.60 ± 0.50, 5.50 ± 0.51, and 2.43 ± 0.50. ∗ indicates obvious difference in NRS scores at *T*_1_ among the three groups (*t* = 10.023, *P* < 0.001). ∗∗ indicate obvious difference in NRS scores at *T*_2_ among the three groups (*t* = 15.645, *P* < 0.001).

**Figure 2:** BCS scores ($\bar{x}\pm s$). The horizontal axis indicates groups A, B, and C, and the vertical axis indicates BCS score (points). The BCS scores of groups A, B, and C were, respectively, 1.15 ± 0.15, 2.36 ± 0.26, and 3.45 ± 0.28. ∗ denotes significant difference in BCS scores between groups A and B (*t* = 22.079, *P* < 0.001); ∗∗ denote significant difference in BCS scores between groups A and C (*t* = 39.659, *P* < 0.001); and ∗∗∗ denote significant difference in BCS scores between groups B and C (*t* = 15.625, *P* < 0.001).

**Table 1:** Clinical data.

	Group A (*n* = 30)	Group B (*n* = 30)	Group C (*n* = 30)	*x* ^2^ or *t*	*P*
Gender (cases)				0.045	0.863
Male	17 (56.67%)	16 (53.33%)	17 (56.67%)		
Female	13 (43.33%)	14 (46.67%)	13 (43.33%)		
Mean age (years)	51.67 ± 5.46	52.70 ± 7.49	53.07 ± 8.45	0.517	0.617
Mean height (cm)	171.97 ± 5.67	167.90 ± 5.72	168.13 ± 6.23	1.805	0.302
BMI (kg/m^2^)	26.85 ± 1.49	26.81 ± 1.35	26.63 ± 1.53	0.385	0.706
Surgery time (min)	66.76 ± 8.99	69.32 ± 9.25	67.39 ± 9.42	0.718	0.500
ASA class (cases)				0.136	0.730
I	12 (40.00%)	13 (43.33%)	14 (46.67%)		
II	18 (60.00%)	17 (56.67%)	16 (53.33%)		
Educational degree (cases)					
Primary school and junior high school	15 (50.00%)	14 (46.67%)	14 (46.67%)	0.044	0.864
Senior high school and junior college	7 (23.33%)	9 (30.00%)	8 (26.67%)	0.171	0.700
College and above	8 (26.67%)	7 (23.33%)	8 (26.67%)	0.059	0.844
Complicating disease (cases)				0.134	0.732
Diabetes	17 (56.67%)	16 (53.33%)	15 (50.00%)		
Hypertension	13 (43.33%)	14 (46.67%)	15 (50.00%)		
Household economy				0.150	0.717
≥3,000 yuan/(month·person)	21 (70.00%)	20 (66.67%)	19 (63.33%)		
<3,000 yuan/(month·person)	9 (30.00%)	10 (33.33%)	11 (36.67%)		
Place of residence (cases)				0.159	0.710
Urban area	20 (66.67%)	21 (70.00%)	22 (73.33%)		
Rural area	10 (33.33%)	9 (30.00%)	8 (26.67%)		

**Table 2:** Onset time and duration ($\bar{x}\pm s$).

Group	*n*	Onset time (min)	Duration (min)
A	30	3.76 ± 0.18	14.37 ± 4.24
B	30	3.08 ± 0.20^∗^	23.38 ± 2.95^#^
C	30	2.41 ± 0.44^∗^	27.88 ± 1.95^#^

Both ∗ and # indicate *P* < 0.001 versus group A.

**Table 3:** Hemodynamic indexes ($\bar{x}\pm s$).

Item		Before SGB			5 min after SGB	
	Group A	Group B	Group C	Group A	Group B	Group C
HR (bpm)	78.83 ± 5.72	77.17 ± 3.56^a^	78.83 ± 4.76^a^	78.73 ± 5.43	78.37 ± 4.77^aa^	77.03 ± 5.49^aa^
SBP (mmHg)	119.30 ± 8.57	115.63 ± 6.70^b^	120.40 ± 6.10^b^	120.53 ± 6.87	119.20 ± 5.63^bb^	121.97 ± 5.29^bb^
DBP (mmHg)	72.23 ± 2.94	71.10 ± 3.07^c^	71.77 ± 3.64^c^	72.77 ± 3.10	71.47 ± 4.28^cc^	71.13 ± 5.06^cc^
SaO_2_ (%)	97.42 ± 1.28	98.07 ± 1.16^d^	98.48 ± 0.95^d^	97.93 ± 1.34	98.63 ± 1.16^dd^	98.83 ± 0.83^dd^

All a, aa, b, bb, c, cc, d, and dd denote *P* > 0.05 versus group A.

**Table 4:** Adverse reaction rates [*n*(%)].

Group	*n*	Pharyngeal discomfort	Hoarseness	Abnormal sensation in the upper limbs	Dizziness	Total incidence rate
A	30	3 (10.00%)	4 (13.33%)	2 (6.67%)	0 (0.00%)	9 (30.00%)^∗^
B	30	3 (10.00%)	5 (16.67%)	3 (10.00%)	2 (6.67%)	13 (43.33%)^#^
C	30	6 (20.00%)	6 (20.00%)	5 (16.67%)	4 (13.33%)	21 (73.33%)

Both ∗ and # denote *P* < 0.05 versus group C.

## Data Availability

Data used to support the findings of this study are available on reasonable request from the corresponding author.
